# Study of PD-1 Customization and Autoimmune T Cells for Advanced Colorectal Cancer with High MSI Expression

**DOI:** 10.1155/2022/6390924

**Published:** 2022-07-31

**Authors:** Na Li, Xiaojie Zhang, Yinsong Zhang, Fang Yang, Fengju Zhou

**Affiliations:** Hengshui City People's Hospital, Hengshui 053000, Hebei, China

## Abstract

**Objective:**

To evaluate the significance of PD-1 customization and autoimmune T-cell therapy for advanced colorectal cancer with high MSI expression.

**Methods:**

One hundred and eight patients with advanced colorectal cancer with high MSI expression admitted to our hospital between August 2019 and January 2022 were divided into control and study groups, and PD-1 customization and autoimmune T-cell therapy were administered to the two groups, respectively. Trends in immune indexes, PD-1 exposure, and survival rates were studied in both groups.

**Results:**

The treatment efficiency of the study group was 90.74%, which was higher than that of the control group (61.11%) (*P* < 0. 05); after treatment, the presence of CDl07a, perforin, and GranB cells was significantly higher in both groups compared with that before treatment, but the expression of PD-1 was more pronounced in the study group (*P* < 0. 05); that is, the expression of PD-1 in peripheral T lymphocytes in the study group compared with that of the control group was higher in patients with grade III-IV, and peripheral T lymphocytes were also higher in patients with grade III-IV compared with patients with grade I-II (*P* < 0. 05).

**Conclusion:**

PD-1 customization combined with autoimmune T-cell therapy is a novel therapeutic modality that can substantially improve.

## 1. Introduction

Nowadays, the society is continuously developing and progressing, people's living habits have changed greatly, and data show that the current incidence of advanced colon cancer is increasing year by year [1]. Patients do not pay great attention to the early stage of the disease, and when they arrive at the hospital for inspection, they are already in the middle and late stage, which delays the best treatment time. In the past, chemotherapy and surgery were mainly used in related practice to improve tumor evolution, but after the treatment, patients experience immunosuppression, which would easily lead to tumor metastasis and recurrence, with poor prognosis and low survival rate [2]. Some patients are contraindicated to undergo surgery since they have immunity system dysfunction, which is not suitable for surgical treatment; so in order to improve the immune function of patients, it is necessary to explore effective ways to lift their immunity status in further studies [3]. Some scholars point out that autoimmune T-cell therapy can be used, but there are few analysis reports on this aspect [4].

In this study, 108 patients with advanced colorectal cancer with high MSI expression admitted from August 2019 to January 2022 were selected, and somatically expanded comprehensive autoimmune cells were infused back into the patients, and the relationship between patient survival and immune function was assessed by several indicators in the hope that this treatment modality will become an important breakthrough for patient prognosis improvement.

The treatment efficiency of the study group was 90.74% higher than that of the control group, that is, 61.11% (*P* < 0. 05); CD4+, CD3+, CD4+/CD8+, CD16+, CD56+, CD4+, and CD25+ in the study group were higher than that of the control group, and CD8+ was lower than that of the control group (*P* < 0. 05); side effects accounted for 42.59% in the study group and 40.74% in the control group, with no significant difference (*P* > 0. 05); the overall survival rate was higher in the study group than in the control group (*P* < 0. 05); Kamofsky score for 1-year survival, 3-year survival, and 5-year survival was higher in the study group than in the control group (*P* < 0. 05); after treatment, the presence of CDl07a, perforin, and GranB cells was significantly higher in both groups than that before treatment, but PD-1 expression in the study group was more pronounced. To provide a safe and novel treatment for patients with advanced colorectal cancer, it is hoped that this treatment can be used as a way to improve patients' prognosis and provide a safe and novel treatment for patients with advanced colorectal cancer.

## 2. Materials and Methods

### 2.1. General Data

One hundred and eight patients with high MSI expression advanced colorectal cancer admitted to our hospital from August 2019 to January 2022 were selected. In the control group (*n* = 54), 31 and 23 cases were male and female, respectively, with mean age (58.32 ± 3.04) years, mean disease duration (4.21 ± 0.27) years, and mean tumor diameter (10.36 ± 1.54) cm; in the study group (*n* = 54), 29 and 25 cases were male and female, respectively, with mean age (59.57 ± 3.07) years and mean disease duration (4.23 ± 0.58). The differences in general information between the two groups were not significant and comparable (*P* > 0. 05).

Inclusion criteria included (1) those diagnosed with high MSI expression advanced colorectal cancer by pathological diagnosis [5]; (2) those with perfect data and knowledge of treatment options; (3) those with expected survival cycle greater than six months; and (4) those with good functional status. Exclusion criteria included (1) those with bone marrow hematopoietic dysfunction; (2) those with hepatic, renal, and cardiopulmonary insufficiency; and (3) lactating or pregnant patients.

### 2.2. Methods

#### 2.2.1. PD-1 Custom Procedure Treatment

Intravenous injection of natalizumab at a dose of 3 mg/kg or 240 mg was given every two weeks until the patient develops unacceptable toxicity or develops disease progression.

#### 2.2.2. Autoimmune T-Cell Therapy

(1) Preparation of immune activated DC-CIK. Collect venous blood, use the Fresenius blood cell separator for centrifugation, use the lymphocyte separator for cell separation and 1 h applanation culture, select the upper nonapplanated cell suspension for CIK preparation, followed by washing of the applanated cells. (2) Preparation of DC. Wash the obtained cells from the previous step to obtain walled cells and culture them in DC complete medium for 24 h. The DC complete medium is replenished on day 3 and 5, respectively, and transfection is performed on day 7 for SOCSl interference adenovirus vector construction. After one day of transfection, the fungus, endotoxin, and bacteria are detected, and if the results were negative, the mature immunoactivated DC is collected and lyophilized in containers. (3) Preparation of CIK. Unsuspended cells are resuspended with patient's autologous plasma and placed in a medium and cultured, and CD3 monoclonal antibody is added after 24 h. Mycobacteria and bacteria are cultured again after 7 d. For cell collection, sterile saline rinses are applied and cell resuspension is performed in 100 ml of own plasma after completion, after which transfusion into patients is done on the 14th and 16th day, respectively.

### 2.3. Observation Indexes

#### 2.3.1. Treatment Effect [6]

Complete disappearance of lesions as CR; no new lesions and 1/2 reduction of original lesions as PR; increase and reduction of original lesions <25% as SD; increase and reduction of lesions >25% as PD; and OR = PR + CR.

#### 2.3.2. Immune Function [7]

Three ml of peripheral blood was drawn, anticoagulated, lymphocyte isolation solution was applied to single nucleated cells, and flow cytometry was applied to detect CD4+, CD3+, CD8+, CD16+, CD56+, and CD25+ in peripheral blood.

#### 2.3.3. Side Effects

Patients were followed up continuously for 6 months to evaluate the occurrence of side effects such as headache, fever, nausea and vomiting, malaise, chills, and muscle pain after treatment.

#### 2.3.4. Overall Survival Rate

Patients were followed up continuously for 5 years, and the survival period was counted for both groups and the mean value was calculated.

#### 2.3.5. Kamofsky Score [8]

0 points: near death or critically ill; 20 points: needing hospitalization, seriously ill; 30 points: bedridden, normal life limited; 40–50 points: needing special care for them, unable to take care of themselves; 60–70 points: can take care of themselves with the assistance of others; 80 points: with obvious symptoms, but able to persist in walking; 90 points: no obvious symptoms, able to live normal life; and 100 points: no symptoms, normal life.

#### 2.3.6. CDl07a, Perforin, GranB Cell Expression [9]

3 ml of peripheral blood was drawn, heparin was anticoagulated, lymphocyte isolation solution was applied to isolate peripheral blood single nucleated cells, and cells were washed using PBS to complete the incubation process. Then flow cytometry was applied to detect the expression of CDl07a, perforin, and GranB.

#### 2.3.7. PD-1 Expression in Peripheral T Lymphocytes

The values of peripheral CD4+ and CD8+ T lymphocytes were counted in the control group, study group, stage I-II, and stage III-IV patients, respectively.

### 2.4. Statistical Methods

Data were analyzed using statistical SPSS 22.0 software, and if the data conformed to normal distribution, the count data were described by composition ratio and rate; and the chi-square test was selected for the analysis of differences between groups, and the measurement data were expressed as (mean ± standard deviation), and the difference was taken to be statistically significant at *P* < 0.05, and the graph software used for the study was GraphPadPrism8.

## 3. Results

### 3.1. Treatment Effect of the Two Groups

The treatment efficiency of the study group was 90.74%, which was higher than that of the control group, 61.11% (*P* < 0.05) (see Table 1).

### 3.2. Comparison of Immune Function between the Two Arms

CD4+, CD3+, CD4+,/CD8+, CD16+, CD56+, CD4+, and CD25+ were higher in the study group than in the control group, and CD8+ was lower than that in the control group (*P* < 0.05). The antibody against BMI-1 and *β*-actin (dilution: 1:1000) was incubated with membranes overnight in the shaker at 4°C. After wash with TBST solution, these membranes were incubated with horseradish peroxidase-conjugated secondary antibody (dilution: 1:1000). Exposure imaging was performed under the Bio-Rad imager, and Image Lab software was used to measure the target band intensities. *β*-actin served as an internal control (see Figure 1).

### 3.3. Comparison of Side Effects between the Two Groups

There was no statutory difference between 42.59% of side effects in the study group and 40.74% in the control group (*P* > 0.05) (see Figure 2).

### 3.4. Comparison of Overall Survival Rate between the Two Groups

The overall survival rate was higher in the study group compared to the control group, and the difference was considered statistically significant when compared between groups (*P* < 0.05) (see Figure 3).

### 3.5. Comparison of Kamofsky Points between the Two Groups

The study group survived 1 year, 3 years, and 5 years corresponding to higher Kamofsky score than the control group (*P* < 0.05) (see Table 2 and Figure 4).

### 3.6. Analysis of CDl07a, Perforin, and GranB Cell Expression in the Two Groups

After treatment, the expression of CDl07a, perforin, and GranB cells in both groups increased significantly compared with that before treatment, but the expression in the study group was more significant (*P* < 0.05) (see Figure 5).

### 3.7. Analysis of PD-1 Expression in Peripheral T Lymphocytes

Compared with the control group, the expression level of PD-1 in peripheral T lymphocytes was higher in the study group, and compared with stage I-II patients, the expression level of PD-1 in peripheral T lymphocytes was higher in stage III-IV patients (*P* < 0.05) (see Figure 6).

## 4. Discussion

Many studies have confirmed that patients with colorectal cancer have the phenomenon of adaptive immunity, and some patients have the phenomenon of intrinsically low function and decreased immune cells [10]. In addition, since the tumor microenvironment of patients with advanced colorectal cancer is prone to immunosuppression and the tumor volume in a relatively large manner, tumor cells are in immunosuppression and resistance after chemotherapy, which is not conducive to the smooth progress of treatment [11]. At present, people's awareness of tumor diseases is getting increasingly high, and it has been recognized that both adaptive immune cells and innate immune cells will participate in the body's antitumor immune process, so they tend to choose autoimmune T-cell therapy [12, 13].

Autoimmune T-cell therapy can restore the number of immune cells in patients, which can improve self-tolerance and resistance and contribute to immune function [14]. In this study, T immune cells were cultured in vitro, which can play an important role in the treatment of viral tumor diseases [15]. In combination with PD-1 custom surgery, nivolumab injection is a fully human monoclonal antibody against the PD-1 receptor and is widely used in locally advanced or metastatic disease. It is an immunologic oncology agent in the treatment of colon cancer [16]. After PD-1 customization of patients, PD-1 receptors expressed in T cells can effectively bind to the ligands PD-L2 and PD-L1, thus inhibiting T-cell factor production and proliferation and at the same time suppressing tumor immunity. Monitoring inhibition can slow down the tumor growth process [17, 18]. Good results were achieved using both of these methods. The results showed that the effective rate of the study group was 90.74%, which was higher than that of the control group, that is, 61.11%. The results confirmed that the combination therapy was more effective compared to a single autoimmune T-cell and PD-1 custom procedure mainly because intravenous infusion of CD3 monoclonal antibodies activates the initial T cells, which in turn induces adaptive immunity [19, 20], and the combination of the two approaches can improve the postoperative survival of patients and minimize the metastasis of tumor cells.

Moreover, an increasing number of studies have confirmed that treatment effects can be predicted by PD-L1 expression [21–23]. The expression level of PD-1 in peripheral T lymphocytes was higher in the study group compared to the control group in this study. Among patients in grades I-II, patients in grades III-IV had higher levels of PD-1 expression in peripheral T lymphocytes [24–26]. Therefore, PD-1 can be used to assess the prognosis of patients, with an increase in CD4+, CD3+, CD16+ CD56+, CD4+ CD25+, and CD8+ after treatment, favoring the improvement of symptoms. The results confirm that PD-1 customized combined with autoimmune T-cell therapy is safe and effective and is a treatment method worth promoting.

In conclusion, PD-1 customized surgery combined with autoimmune T-cell therapy is a new treatment method, which can greatly improve the patient's immune function, prolong the patient's survival period, and the patient's prognosis is good.

## Figures and Tables

**Figure 1:** Immune function in both groups.

**Figure 2:** Two sets of side effects.

**Figure 3:** Overall survival rate in both groups.

**Figure 4:** Two Kamofsky points.

**Figure 5:** Expression of CDl07a, perforin, and GranB cells in two groups.

**Figure 6:** Analysis of PD-1 expression in peripheral T lymphocytes.

**Table 1:** Treatment effect in both groups (*n*, %).

Group	Number of cases	CR	PR	SD	PD	OR
Control group	54	19 (35.19)	14 (25.93)	6 (9.38)	15 (27.78)	33 (61.11)
Study group	54	31 (57.41)	18 (33.33)	3 (5.56)	2 (3.70)	49 (90.74)
X^2^	—	—	—	—	—	12.968
P	—	—	—	—	—	˂0.001

**Table 2:** Comparison of Kamofsky points between two groups.

Score	Research group			Control group		
	Survival of one year	Survival of three years	Survival of five years	Survival of one year	Survival of three years	Survival of five years
100	27.78 (15/54)	15.79 (6/38)	20.00 (1/5)	5.56 (3/54)	9.09 (1/11)	0.00 (0/3)
80	14.81 (8/54)	7.89 (3/38)	0.00 (0/5)	3.70 (2/54)	9.09 (1/11)	33.33 (1/3)
60	9.26 (5/54)	5.26 (2/38)	20.00 (1/5)	1.85 (1/54)	0.00 (0/11)	0.00 (0/3)
40	11.11 (6/54)	5.26 (2/38)	20.00 (1/5)	3.70 (2/54)	9.09 (1/11)	0.00 (0/3)
20	5.56 (3/54)	5.26 (2/38)	20.00 (1/5)	3.70 (2/54)	0.00 (0/11)	33.33 (1/3)

## Data Availability

The experimental data used to support the findings of this study are available from the corresponding author upon request.

## References

[1] Yang W., Lei C., Song S. (2021). Immune checkpoint blockade in the treatment of malignant tumor: current statue and future strategies. *Cancer Cell International*.

[2] Li H., Yang C., Cheng H., Huang S., Zheng Y. (2021). CAR-T cells for Colorectal Cancer: target-selection and strategies for improved activity and safety. *Journal of Cancer*.

[3] Ahlmanner F., Sundström P., Akeus P. (2018). CD39+ regulatory T cells accumulate in colon adenocarcinomas and display markers of increased suppressive function. *Oncotarget*.

[4] Bashir B., Flickinger J. C., Snook A. E. (2021). Vaccines and immune checkpoint inhibitors: a promising combination strategy in gastrointestinal cancers. *Immunotherapy*.

[5] Masucci G. V., Cesano A., Hawtin R. (2016). Validation of biomarkers to predict response to immunotherapy in cancer: volume I—pre-analytical and analytical validation. *Journal for immunotherapy of cancer*.

[6] Pao W., Ooi C. H., Birzele F. (2018). Tissue-specific immunoregulation: a call for better understanding of the “immunostat” in the context of cancer. *Cancer Discovery*.

[7] Santarpia M., Aguilar A., Chaib I. (2020). Non-small-cell lung cancer signaling pathways, metabolism, and PD-1/PD-L1 antibodies. *Cancers*.

[8] Sorrentino C., D’Antonio L., Fieni C., Ciummo S. L., Di Carlo E. (2021). Colorectal cancer-associated immune exhaustion involves T and B lymphocytes and conventional NK cells and correlates with a shorter overall survival. *Frontiers in Immunology*.

[9] Chen Y., Li Y., Guan Y. (2020). Prevalence of PRKDC mutations and association with response to immune checkpoint inhibitors in solid tumors. *Molecular oncology*.

[10] Harada K., Kaya D. M., Song S., Baba H., Ajani J. A. (2017). Genomic profiling of colorectal cancers and the future of personalized treatment. *Colorectal Cancer*.

[11] Wu Z., Li S., Zhu X. (2021). The mechanism of stimulating and mobilizing the immune system enhancing the anti-tumor immunity. *Frontiers in Immunology*.

[12] Golkaram M., Salmans M. L., Kaplan S. (2021). HERVs establish a distinct molecular subtype in stage II/III colorectal cancer with poor outcome. *NPJ genomic medicine*.

[13] Schlößer H. A., Thelen M., Lechner A. (2019). B cells in esophago-gastric adenocarcinoma are highly differentiated, organize in tertiary lymphoid structures and produce tumor-specific antibodies. *OncoImmunology*.

[14] Yarchoan M., Johnson B. A., Lutz E. R., Laheru D. A., Jaffee E. M. (2017). Targeting neoantigens to augment antitumour immunity. *Nature Reviews Cancer*.

[15] Reichert Z. R., Urrutia J., Alumkal J. J. (2019). Microsatellite instability as an emerging biomarker for checkpoint inhibitor response in advanced prostate cancer. *JAMA Oncology*.

[16] Granier C., Gey A., Roncelin S., Weiss L., Paillaud E., Tartour E. (2021). Immunotherapy in older patients with cancer. *Biomedical Journal*.

[17] Le Louedec F., Leenhardt F., Marin C., Chatelut É., Evrard A., Ciccolini J. (2020). Cancer immunotherapy dosing: a pharmacokinetic/pharmacodynamic perspective. *Vaccines*.

[18] Kanygina A. V., Sharova E. I., Sultanov R. I. (2019). Targeted gene sequencing panels: applicability for neoantigen profiling of colon and rectal adenocarcinoma. *Biochemistry (Moscow), Supplement Series B: Biomedical Chemistry*.

[19] Ajina A., Maher J. (2019). Synergistic combination of oncolytic virotherapy with CAR T-cell therapy. *Progress in Molecular Biology and Translational Science*.

[20] Chabanon R. M., Rouanne M., Lord C. J., Soria J. C., Pasero P., Postel-Vinay S. (2021). Targeting the DNA damage response in immuno-oncology: developments and opportunities. *Nature Reviews Cancer*.

[21] Bruno V., Corrado G., Baci D. (2020). Endometrial cancer immune escape mechanisms: let us learn from the fetal–maternal interface. *Frontiers in Oncology*.

[22] Guven D. C., Sahin T. K., Erul E., Kilickap S., Gambichler T., Aksoy S. (2022). The association between the pan-immune-inflammation value and cancer prognosis: a systematic review and meta-analysis. *Cancers*.

[23] Stroncek D. F., Butterfield L. H., Cannarile M. A. (2017). Systematic evaluation of immune regulation and modulation. *Journal for ImmunoTherapy of Cancer*.

[24] Huang X., Tang T., Zhang G. (2020). Genomic investigation of co-targeting tumor immune microenvironment and immune checkpoints in pan-cancer immunotherapy. *NPJ precision oncology*.

[25] Merritt C. R., Ong G. T., Church S. E. (2020). Multiplex digital spatial profiling of proteins and RNA in fixed tissue. *Nature Biotechnology*.

[26] Affolter A., Kern J., Bieback K., Scherl C., Rotter N., Lammert A. (2022). Biomarkers and 3D models predicting response to immune checkpoint blockade in head and neck cancer. *International Journal of Oncology*.

